# Analysis of Regional Economy Development on Local Environmental Protection and Natural Resources Utilization from the Perspective of Big Data

This article has been retracted.

**DOI:** 10.1155/2022/9461377

**Published:** 2022-09-29

**Authors:** Yuanzhang Wen

**Affiliations:** School of Economics, Sichuan University, Chengdu, 610065 Sichuan, China

## Abstract

The ecological restoration and civilization construction is one of the key tasks in China. The economic development of different regions has different effects on the resource protection and utilization. In the face of complex natural conditions and resource-rich areas, how to carry out the ecological environment promotion work is put forward. The urbanization level of the Yangtze River region increases from 17.9% to 60.6%, showing the characteristics of rapid expansion. In the face of urban diseases such as unreasonable industrial layout, it is urgent to improve regional economy and promote green urban development from the perspective of big data. Adhering to the concept of ecological priority, the development of digital technology drove the development of local economy in 2019, accounting for 43% of the national population. While promoting the economic development, it is of great significance to ensure the efficiency of resource utilization and promote the high-quality development of common economy.

## 1. Introduction

Urban green transformation is to develop within the carrying capacity of economy, society and environment, realize green production mode, green lifestyle, and inclusive social environment, and promote the city to take the road of intensive, intelligent, and beautiful ecology. It can be seen that the concept of “green transformation” has a strong consistency with the goal of “production-living-ecological” space optimization in connotation, that is, to promote intensive and efficient production space, livable, and moderate living space, and beautiful ecological space. As an advanced form of economic and social development, digital economy strengthens the integration of urban development and industrial development from the perspective of big data, plays an important role in industrial transformation and upgrading, social governance, and other fields. And it gradually becomes a new driving force leading the green transformation and development of cities. It is of great significance to further exert the development of digital economy to lead the green transformation of cities and boost the high-quality development of cities. Urban agglomeration is the highest form of spatial organization in the mature stage of urban development. It refers to a specific region with at least one megalopolis as its core and at least three large cities as its units. Relying on the developed infrastructure network such as transportation and communication, it forms a city group with compact spatial organization and close economic connection, and finally realizes the high degree of integration. Urban agglomeration is a large, multicore and multilevel city group formed by a number of geographically concentrated megacities and big cities, which is the union of metropolitan areas. At present, there are six world-class urban agglomerations universally recognized around the world: the Atlantic coastal urban agglomerations in the northeast of the United States, the Great Lakes urban agglomerations in North America, the Pacific coastal urban agglomerations in Japan, the British urban agglomerations in the northwest of Europe, and the Yangtze River Delta urban agglomerations. Urban agglomeration will be the most dynamic and potential strategic support and growth pole in China's future economic development pattern and dominate the lifeblood of national economic development. As a link of regional economic and social connection, transportation is a necessary guarantee for the formation and development of urban agglomerations. Meanwhile, the layout of transportation facilities will also affect the spatial structure and evolution mode of urban agglomerations. Since the reform and opening up, China's urban agglomeration and regional transport system has been constantly mature, the quality of transport facilities and transport mileage has been constantly improved. At present, all urban agglomerations in China have formed relatively perfect high-speed transportation systems, which play an important driving role in the spatial conduction and effective allocation of inter-city production factor flow and the optimization and reorganization of urban agglomerations spatial structure, as shown in Figure 1.

Transportation integration is an important support and guarantee for the implementation of regional coordinated development strategy and national development strategy of Yangtze River Delta regional integration. In particular, high-speed transportation system can produce many linkage development effects and is an important driving force for shaping urban gateway effect and efficient utilization of resources. On September 19, 2019, the Outline of Building China into a Transport Country issued by the CPC Central Committee and The State Council clarified the development goal of “basically building China into a transport country by 2035 and comprehensively building China into a transport country that is satisfactory to the people and at the forefront of the world by the middle of the 21st century”. At the end of 2019, the Outline of the Plan for regional Integrated Development of the Yangtze River Delta defined the transportation tasks of “jointly building the Yangtze River Delta on the track”. Although the construction of high-speed transportation system in the Yangtze River Delta region has a good foundation for development, it still faces some bottleneck problems, such as unbalanced development of high-speed transportation system, uncoordinated high-speed transportation subsystem and the overall competitiveness of transportation to be improved. Therefore, it is necessary to put the construction of high-speed transportation into the overall regional integration development of the Yangtze River Delta, and fully realize the role of high-speed transportation in the implementation of the integration strategy of the Yangtze River Delta, as shown in Figure 2.

In recent years, China's international and domestic tourism income has achieved fruitful results. The tourism performance and tourism market are well-developed. However, with the advent of the era of mass tourism, some quality shortcomings in the development of China's tourism industry are gradually exposed. For example, the insufficient tourism products effective supply cannot adapt to the people's growing travel demand. The imbalance of urban and rural tourism development cannot adapt to the global tourism development. The insufficient novelty of tourism product forms cannot adapt to individuation and diversification of tourism consumption demand. The tourism theory research cannot adapt to the rapid development of tourism industry practice. The huge tourism economies are not coordinated with the low operational efficiency of tourism industry. With the fragmentation of the tourism market of consumer demand and multiple overlays is forming, if China's tourism industry cannot improve, transform, and innovate in terms of supply side, demand side, and industrial operation efficiency in a timely manner, it may be difficult to jump out of the “primary stage of mass tourism trap”. If it follows the trend of great changes unseen in the world and high-quality economic development, the tourism industry will enter a new blue ocean, as shown in Figure 3.

## 2. Literature Review

On the basis of systematic review and summary of relevant domestic and foreign research literature, a theoretical research framework is built based on tourism destination system theory, traffic economic belt theory, coupled and coordinated development theory, and unbalanced development theory of regional economy in the research. Following the research line of theoretical model construction of high-speed traffic dominance degree, tourism intensity, and their coupling coordination → comprehensive score calculation of high-speed traffic dominance degree and tourism intensity → verification of the spatiotemporal dynamic relationship between high-speed traffic dominance degree and tourism intensity → grasping the evolution law and simulating the trend prediction of spatio-temporal coupling coordination degree of high-speed traffic dominance degree and tourism intensity → revealing the influence mechanism of the spatiotemporal evolution of the coupling coordination degree of the high-speed traffic dominance degree and the tourism intensity → proposing the optimal path and policy suggestions for the coupling coordination between the high-speed transportation dominance degree and the tourism intensity, integrating multiple comprehensive evaluation model, coupling coordination model, Arc GIS spatial analysis technology, mathematical statistics analysis technology, spatial econometric model and multiple method model, the spatio-temporal evolution, and multidimensional driving mechanism of transport and travel coupling coordination degree in the Yangtze River Delta are systematically investigated. The specific research ideas are as follows:first, it is based on theoretical model construction and comprehensive development level calculation of geographical elements [1]. On the basis of constructing the theoretical evaluation model framework of high-speed traffic superiority degree and tourism intensity, the mathematical statistics methods, such as entropy weight TOPSIS method, Bootstrap-DEA model, box graph and kernel density curve, and Arc GIS spatial analysis technology are used to measure the high-speed traffic superiority degree and tourism intensity of cities in the Yangtze River Delta region. The respective time series evolution characteristics of the Yangtze River Delta regional scale, provincial scale and prefecture-level city-scale high-speed traffic dominance degree and tourism intensity theory are explored, and the evolution types of prefecture-level city-scale high-speed transportation dominance degree and tourism intensity are refined. ArcGIS spatial analysis technology is used to measure the spatial and temporal differentiation characteristics of high-speed traffic dominance and tourism intensity, which is the basic work for the follow-up in-depth research of the thesis.

The range standardization method is used for data processing, and the normalized index matrix is multiplied by the weight matrix determined by the entropy weight method to obtain the weighted normalized evaluation matrix *Y*, as shown in

(1) $$\begin{array}{c} Y=\left[\begin{array}{cccc} Y_{11} & Y_{12} & \cdots & Y_{1m}\\ Y_{21} & Y_{22} & \cdots & Y_{2m}\\ \cdots & \cdots & \cdots & \cdots \\ Y_{n1} & Y_{n1} & \cdots & Y_{nm} \end{array}\right]=\left[\begin{array}{cccc} r_{11}\cdot \omega_{1} & r_{12}\cdot \omega_{2} & \cdots & r_{1n}\cdot \omega_{n}\\ r_{21}\cdot \omega_{1} & r_{22}\cdot \omega_{2} & \cdots & r_{2n}\cdot \omega_{n}\\ \cdots & \cdots & \cdots & \cdots \\ r_{m1}\cdot \omega_{1} & r_{m2}\cdot \omega_{1} & \cdots & r_{mn}\cdot \omega_{n} \end{array}\right]. \end{array}$$

In Formula (1), rmn represents the *n*th index in the *m*th year after standardization, and *ω* refers to weight. Positive and negative ideal solutions are determined as.

(2) $$\begin{array}{c} \begin{array}{c} Y^{+}=\max\left\{\left(y_{\text{ij}}\left|\text{i}=1,2,\cdots ,m\right.\right)\right\}\left(j=1,2,\cdots ,n\right)=\left\{y_{1}^{+},y_{2}^{+},\cdots ,y_{\text{n}}^{+}\right\},\\ Y^{‐}=\min\left\{\left(y_{\text{ij}}\left|\text{i}=1,2,\cdots ,m\right.\right)\right\}\left(j=1,2,\cdots ,n\right)=\left\{y_{1}^{-},y_{2}^{-},\cdots ,y_{\text{n}}^{-}\right\}. \end{array} \end{array}$$

In Formula (2), *Y*^+^ represents the maximum value of the *j*th index in the year *i*, and *Y*^+^ is the positive ideal solution, which can be selected as the most ideal scheme. *Y*^−^ represents the minimum value of the *j*th index in the year *i*, and *Y*^−^ is the negative ideal solution, namely the worst scheme [2], as shown in Figure 4.

The second is based on the verification of the spatial-temporal dynamic relationship between high-speed traffic dominance and tourism intensity. Determining the spatio-temporal dynamic relationship between the superiority degree of high-speed transportation and tourism intensity and the degree of interaction is a prerequisite for calculating the coupling coordination degree of transportation and tourism [3]. Bivariate LISA model, decoupling effect model, and panel vector autoregressive model are used to verify the spatio-temporal dynamic relationship between high-speed transportation superiority and tourism intensity from different perspectives of spatio-temporal correlation effect, decoupling effect, and dynamic interaction effect.

The third is to grasp the spatial and temporal evolution characteristics of the coupling coordination degree of high-speed transportation superiority and tourism intensity at multiple scales and from multiple perspectives and predict its future development trend. Based on the coupling coordination degree model, Arc GIS trend surface analysis module, Exploratory spatial Data analysis (ESDA), standard Deviation ellipse model (SDE), LISA time path and temporal, and spatial transition analysis (ESTDA) are used to calculate the coupling coordination index of high-speed transportation superiority and tourism intensity. The spatio-temporal evolution of the coupling coordination degree of high-speed traffic superiority and tourism intensity in the Yangtze River Delta region is studied from the perspectives of overall trend, spatial differentiation, spatial correlation, pattern evolution, and spatio-temporal dynamic evolution path [4]. The modified grey forecasting GM (1, 1) model is used to predict and simulate the future development level of coupling coordination degree between highway traffic superiority degree and tourism intensity in 41 cities in the Yangtze River Delta region. From the global perspective, the temporal and spatial trends of the future coordinated development of high-speed transportation construction and tourism development in the Yangtze River Delta region are analyzed.

The fourth is to scientifically reveal and systematically refine the driving mechanism of the spatio-temporal evolution of the coupling coordination degree between the superiority degree of high-speed transportation and tourism intensity, and put forward the optimization strategy of the integration of transportation and tourism [5]. Firstly, influence variables with internal and external layers are constructed based on multisource heterogeneous data, and ridge regression analysis method, panel quantile regression model (Figure 5), system dynamic panel regression model (SGMM), and spatial panel econometric model are comprehensively adopted. From the perspectives of internal endogenous force, interaction influence and external driving force, the internal action mechanism, interaction influence mechanism, and external driving mechanism of the spatio-temporal evolution of the travel-travel coupling coordination degree in the Yangtze River Delta region are extracted, respectively. The effect process, intensity and nature of each variable on the change of travel-travel coupling coordination degree in the Yangtze River Delta are systematically analyzed, and the main driving forces affecting the spatial differentiation of travel-travel coupling coordination degree are clarified [6]. Secondly, according to a series of empirical research conclusions, as well as the actual situation of high-speed transportation construction and tourism development in the Yangtze River Delta region, the optimization path and policy suggestions are proposed to promote the coupling and synergistic development of high-speed transportation superiority degree and tourism intensity in the Yangtze River Delta region. It provides an important basis for the construction of high-speed transportation system and the decision of regional tourism spatial integration and optimization in Yangtze River Delta.

## 3. Research on the Interactive Relationship between High-Speed Transportation System and Tourism Development

Some scholars' studies have shown that aircraft have the largest nitrogen oxide and carbon dioxide emissions, the highest energy demand and environmental cost, and buses have the highest nitrogen and hydrogen compounds emissions [7]. In (Table 1), railway transportation has a good effect in all classification investigations. Some scholars found that the waste emissions in Hainan increased under the operation of high-speed rail, as shown in Figure 6.

### 3.1. Theory of Regional Unbalanced Development

#### 3.1.1. Regional Pole Theory

French economists formally put forward the concept of “growth pole” in the article On the Concept of “Growth Pole”. In 1966, French geographer defined “growth pole” as the industrial complex with expanding urban area configuration and guiding the further development of economic activities under its influence. Growth pole is the “engine” of regional social activities and economic growth, which can form a polar core spatial structure. Later, on this basis, economic geographer Miller and Kiernan proposed the theory of “dual-core” spatial structure according to the development reality of China's coastal and riverside areas [8], as shown in Figure 7.

According to the growth pole theory, the backward regions are generally broad in area and rich in natural resources, but these regions tend to have poor natural conditions, low degree of development, weak economic foundation, low transportation accessibility, and poor investment environment, etc., which seriously lack central cities to drive the overall development of the region. In this case, in order to accelerate the economic development of the above regions, the key is to cultivate the rise of central cities that can drive the overall development of the region and implement the unbalanced development strategy [9]. There are two ways to form the growth pole. One is to realize the agglomeration of factors of production in large central cities by using the mechanism of market spontaneous regulation, and give play to its agglomeration and scale effect to form the regional growth pole. The second is to give full play to the government's macrocontrol role and use the government's intervention role. Adhering to the concept of “concentrated investment, key construction, agglomerated development, focusing on diffusion”, regions, and industries with better conditions are selected to give key support and large-scale economic growth poles are cultivated, so as to give full play to the linkage role of the growth pole of “point to surface”, as shown in Figure 8.

The tourism growth pole accelerates or restrains the tourism in the surrounding areas mainly through its polarization and diffusion. On the one hand, the polarization of tourism growth pole will lead to the gap of tourism development strength between it and its neighboring regions. On the other hand, by exerting its scale and agglomeration effect, tourism growth pole can transfer its tourism information flow, talent flow, capital flow, and tourism flow to the adjacent areas, and then play a driving role in the development of tourism in the adjacent areas. To a certain extent, it enlarges the tourism connection intensity among the tourism nodes and makes the node tourism economic connection model tend to compound network. At the same time, the tourism growth pole theory also provides useful theoretical guidance for less developed tourism areas to develop core tourism nodes by centralizing superior resources through government macrocontrol policies and exerting the regional linkage effect of tourism core nodes on surrounding cities, as shown in Figure 9.

The quality and radiation range of tourism nodes have also expanded significantly. Tourism exchanges and connections between tourism nodes must be supported by the transportation network system, which puts forward higher requirements for the quality and scale of transportation construction (axis). That is, the tourism axis between the nodes will gradually penetrate vertically and horizontally, thereby forming a set of tourism connection networks between multiple nodes. In a word, in the “point-axis” system theory of regional tourism destination, its basic elements include tourism nodes, tourism transportation axis, and tourism element flow [10]. The difference in development strength and industrial structure among tourism nodes is the internal dynamic mechanism for the formation of their agglomeration and diffusion effects. The tourism development axis is the bridge and carrier of the spatial transmission and configuration of the development factor flow between tourism nodes. Tourism element flow is the material and nonmaterial medium of spatial interaction between tourism nodes, as shown in Figure 10.

### 3.2. Construction of the Coupling Collaborative Evaluation Model of High-Speed Traffic Superiority Degree and Tourism Intensity

The construction of “transport-travel” collaborative evaluation model is the basic work to calculate the coupling coordination degree of high-speed transportation superiority degree and tourism intensity. In the past, few studies have constructed the collaborative evaluation model of the two, which is not conducive to the understanding of the connotation of the coordination degree of transport and travel coupling and the systematic disclosure of its evolution law. High-speed transportation system and urban tourism development have a coupling and synergistic development trend and dynamic interaction process in geographical space, and this trend and process often promote the synergistic effect of transportation and tourism in physical space and virtual space, showing the continuous improvement of the coupling coordination level of transportation and tourism [11]. It is difficult to find an accurate model to evaluate these coupling synergistic relationships. In order to solve this problem, a more flexible evaluation system is needed to analyze the coordination process of “transport-travel”, as shown in Figure 11.

The relationship between high-speed traffic advantage degree and intensity of tourism space coupling coordination degree (D), tourism intensity (TI), and high-speed traffic dominance (HST) is not a simple linear, but reflects the process of mutual optimization and integration and reorganization between systems [12]. It is the continuous process of driving reconstruction, mutual integration, and configuration optimization of the intersystem element system that can promote the coupling synergistic effect of high-speed transportation superiority and tourism intensity from low level (extreme imbalance) to high level (excellent coordination), as shown in Figures 12–14.

## 4. Thoughts and Suggestions on the Development of Regional Tourism Towns

### 4.1. Urban Products

With the continuous advancement of China's urbanization process, the level of urbanization has been significantly improved. The urbanization rate is increasing year by year, the construction of urban public infrastructure is improving day by day, and the supply level and capacity of urban public services have been improved to some extent. People enjoy a certain sense of gain and happiness [13]. However, there is no denying that there are also some problems in big cities, such as traffic congestion, shortage of education and medical resources, environmental pollution, group anxiety caused by stylized life pace, great psychological pressure of residents in big cities, and the proportion of people in subhealth state is increasing. On the whole, China's production capacity of modern industrial products has increased, while the supply capacity of ecological products has weakened, as shown in Figure 15.

With the improvement of people's income level and living standard, the demand for fresh air, clean water, pleasant climate, and other ecological products, as well as the demand for leisure and health care seeking spiritual “habitat” and relieving pressure of tourism consumption is increasing day by day. An important reason for the sustainable development of small tourism towns in ethnic minority areas in the upper reaches of Minjiang River lies in the fact that this region can produce and provide characteristic products and play special functions. Relying on the huge population volume of Chengdu-Chongqing urban agglomeration, it forms normal complementarity and communication with the products and functions provided by the large urban agglomeration. In other words, the region offers specific products and features that people in big cities need. Correspondingly, products such as strong and diverse ideas, advanced technological equipment, advanced concepts, convenient official service products, and huge consumer groups infused with postmodern consumer culture in big cities are urgently needed for the development of the region. The two products and functions can complement each other, so as to achieve the continuous dynamic optimization in mutual promotion [14], as shown in Table 2.

### 4.2. Product Relationship between Regional Tourism Towns and Large Urban Agglomerations

Tourism small towns in ethnic minority areas in the upper reaches of Minjiang River connect the vast rural hinterland of the region with large urban agglomerations. Based on high-quality characteristic natural tourism resources, they produce and provide high-quality tourism products covering happiness industries. Relying on Chengdu-Chongqing urban agglomerations, they radiate to major urban agglomerations in southwest China and even the whole country. It can meet the needs of people in large urban agglomerations for food safety, green ecological agricultural products, parent-child education, ethnic culture with different characteristics, handicrafts of minority ethnic groups, and other aspects [15]. It is complementary to the products produced and provided by the large urban agglomeration, and the two have formed perfect and regular complementarity in terms of products and functions. The tourism towns in this region and the Chengdu-Chongqing urban agglomeration present their own continuous optimization and upgrading situation through two-way complementarity of products, which promotes the innovation and upgrading of tourism products and the development of tourism industry structure in this region, as well as the economic and social development and the sustainable development of tourism towns in this region. The complementary relationship between the two is shown in Figure 16.

The supply-side structural reform of tourism in ethnic minority areas in the upper reaches of Minjiang River should be actively promoted to improve the supply system structure and quality of tourism products in the region, so as to consolidate the industrial foundation for the sustainable development of small tourism towns in the region. Continuous tourist flow is the fundamental guarantee for the sustainable development of small tourist towns, and the continuous innovation and development of tourism products and their characteristics is the key to attract tourists. The upgrading of tourism product structure and the continuous improvement of tourism product quality are the foundation of the upgrading of tourism industry structure. Due to the inertia of tourism industry, minority areas in the upper reaches of Minjiang River fail to timely adapt to the consumer demand of independent personalized tourism era, and the concept and quality of the main body of the product supply system lag behind the changing trend of consumer demand of tourists for a long time, which affects and restricts the sustainable development of tourism economy in this region [16]. Therefore, it is necessary to innovate and upgrade the supply system of tourism products in this region, so as to promote the innovation and upgrade of tourism industry in this region and consolidate the industrial foundation of tourism towns in this region. Tourism products have obvious characteristics of simultaneous production and consumption and nontransferability, which makes the location conditions and accessibility of tourist destinations become important factors affecting the development of tourism in ethnic areas. The natural and cultural tourism resources and ethnic cultural resources of tourist destinations affect the location conditions to a great extent. The small tourist towns in ethnic minority areas in the upper reaches of the Minjiang River should, based on their own resources and functional positioning, conduct in-depth analysis and research on the characteristics and evolution trends of the individual, differentiated, and autonomous travel consumption demands of consumer groups under the influence of postmodern consumer culture, and implement differentiated tourism development. The strategy focuses on the regional complementarity of the tourism product supply system and the differentiated supply of tourism products, promotes the complementarity, and sharing of tourism resources among small tourist towns, realizes the coordinated development of small tourist towns, and forms a regional tourism development community, as shown in Figure 17.

Culture and tourism are like poetry and distance. People's consumption level is constantly improving with the increase of income level; the same is true of tourism consumption. At first, it is the popular tourism consumption level, and with the cultural level of mass tourists, the tourism consumption level is increasing to the cultural consumption level. Visitors enter the new normal economic development; tourism consumption groups gradually show a trend of younger, self-independence, and individuation. The function elements in tourism are also greatly expanded and improved [17]. People pay more attention to the individuation of the travel experience and identity, group identification function. Therefore, the supply of personalized experiential tourism products can not only meet people's basic consumption needs for tourism to achieve the function of tourists' leisure and entertainment but also drive tourists to personalize tourism experience to achieve the purpose of “experience it with the body and experience it with the heart” [18]. It can also promote tourists to consume personalized experience tourism products, realize the function of tourist group identification and identity identification, and maximize the expansion functions and benefits of tourism. In addition, when planning and designing small tourist towns in the region, the differentiated national culture of the region should be integrated with modern architectural technology and art, and the special identification of national culture should be integrated into the urban construction. Combined with the regional natural environment, thematic image, and the characteristics of national culture, the planning and construction of urban characteristic cultural blocks, architectural styles, etc., implementing the concept of global tourism, the characteristic architecture, culture, and art of the local ethnic group are fully demonstrate to make the ethnic characteristic architecture and urban landscape become an important part of the attractiveness and brand image of small tourist towns [19, 20], as shown in Figure 18.

## 5. Conclusions

Excellent natural ecological environment is an important environmental support for the development of tourism. Excellent natural ecological environment itself is tourism resources, which can be developed into tourism products and extend the industry chain of tourism industry. At the same time, it can serve as environmental support for other tourism products, provide benign development space for the development of tourism in the region and the construction of tourism towns, and participate in the production and supply of tourism products in the region, becoming an important part of the tourism product system in the region. Therefore, it is necessary to strengthen ecological environment protection and environmental restoration in minority areas of the upper reaches of Minjiang River to provide environmental support for the development of tourism towns in this area. Building unique and outstanding traditional culture based on regional economy is abundant resources in national regions of the upper reaches of Minjiang river, the continuous culture source power of the region's tourism product innovation and development, the source of the core of the regional tourism products attractive tourism in the construction of small towns in the region, and the cultural source of highlighting its local characteristics. For the innovation and upgrading of tourism products, the sustainable development of tourism industry and the continuous promotion of tourism small towns in this region, the advantage resources of ethnic characteristic culture must be grasped, which has the most vitality. The stability and harmony of soft environment in minority areas in the upper reaches of Minjiang River depends on the effect of social governance. A stable and harmonious social environment is the social guarantee for the steady development of tourism in this region and the continuous promotion of tourism towns. The development of tourism depends on a safe and stable social environment. With the development of tourism in ethnic areas, a large number of tourists flood in, resulting in a variety of contradictions and disputes due to cultural differences, conflicts of interests, and other reasons. The uneven distribution of benefits brought by the development of tourism economy also leads to the increase of contradictions among the people in small tourist towns. If this situation is not managed well, it will inevitably affect the sustainable development of tourism in this region and the healthy development of tourism towns.

Rural revitalization and new-type urbanization, the two national strategies will have a significant impact on the economic and social development of China's rural areas, especially the ethnic minority areas in the upper reaches of the Minjiang River for a long period of time. Therefore, small tourist towns in this region, as well as economic and social development, national culture protection and inheritance, and rural grass-roots governance are research hotspots and directions for further research in this region. The research is expected to make due contributions to the economic and social development of the region. In view of the insufficient application of measurement methods in the research, it will continue to be improved according to my own actual situation, so as to conduct an in-depth research on the region.

## Figures and Tables

**Figure 1:** Basic situation of China's high-speed railway development.

**Figure 2:** Basic situation of China's expressway mileage and civil aviation route mileage.

**Figure 3:** The tourism development in China.

**Figure 4:** Evolution mode of spatial structure.

**Figure 5:** Schematic diagram of regression model in high-speed traffic system.

**Figure 6:** Research framework system of traffic clearance relationship.

**Figure 7:** Tourism system.

**Figure 8:** Development stages of traffic economic belt.

**Figure 9:** Schematic diagram of polarization mode.

**Figure 10:** Evolution of the “point-axis” spatial structure system.

**Figure 11:** Theoretical logic of the internal relationship between high-speed traffic and tourism intensity and its subsystems.

**Figure 12:** Construction of coupling coordination degree evaluation model.

**Figure 13:** Conceptual model of strength.

**Figure 14:** Demand intensity evaluation model.

**Figure 15:** Time change of the comprehensive evaluation index of high-speed traffic dominance degree.

**Figure 16:** Complementary products of tourism small towns and large urban agglomerations in the upstream ethnic regions.

**Figure 17:** Regional tourism industry development and tourism town development.

**Figure 18:** Cultural inheritance and protection and tourism development.

**Table 1:** Comparison of impacts of different modes of tourism transportation on tourism environment.

The image content	Private cars	Buses	Civil aviation	Trains
HC (threat to health)	0.01	0.05	0.03	0
CO (threat to health)	0.19	0.05	0.13	0
NOx (acid rain formation)	0.06	0.30	0.38	0
CO_2_ (greenhouse effect)	67.3	17.53	105.11	0.9
Energy consumption (KWH)	250	66	409	42
Environmental costs (SEK)	28.11	19.32	42.02	0.38

**Table 2:** Descriptive statistical results of variables.

The variable name	Numbers of samples	Average	Standard deviation	Minimum value	Maximum value
Urban green transformation	880	0.115	0.017	0.074	0.207
Ecological space transformation	880	0.090	0.040	0.021	0.0642
Level of economic development	880	0.242	0.106	0.038	0.759
Technological innovation level	880	1.407	1.427	0.020	15.977
Level of urbanization	880	53.072	12.858	22.600	89.600

## Data Availability

The labeled data set used to support the findings of this study is available from the corresponding author upon request.
